# Effects of mir-195 Targeted Regulation of JAK2 on Proliferation, Invasion, and Apoptosis of Gastric Cancer Cells

This article has been retracted.

**DOI:** 10.1155/2022/5873479

**Published:** 2022-07-26

**Authors:** Yu Zhang, Kun Zhuang, Shanshan Yuan, Wangli Si, Yijun Li, Jun Zhang, Jiaming Liu

**Affiliations:** Department of Gastroenterology, Xi'an Central Hospital, Xi'an, 710003 Shaanxi, China

## Abstract

**Background:**

Overexpression of miR-195 can make gastric cancer cells stay in G1/G2 phase. miR-195 has been shown to inhibit gastric cancer cell replication and accelerate cell death by targeting JAK2. However, the relationship between miR-195, JAK2, and gastric cancer is not clear.

**Objective:**

To observe the effect of mir-195 regulated by JAK2 on the growth, invasion, and death of gastric cancer cells.

**Methods:**

MGC803 and NCI gastric N87 cells were introduced into the negative control sequences of miR-195 and RNA, respectively. To detect the expression of miR-195 in cells, to detect the effect of miR-195 on mitosis and proliferation of tumor cells, to analyze the effect of miR-195 on cell invasion and metastasis, and to detect the regulation of miR-195 on JAK2 expression.

**Results:**

The level of miR-195 in miR-195-MIMICS group was significantly higher than that in miR-NC group. The cell survival rate of miR-195 mimic group was lower than that of miR-NC group (*P* < 0.05). Compared with miR-NC group, the number of cells in G1 phase increased, the cells in G2 phase and S phase decreased, and the proportion of cells in G2 and S phase decreased in miR-195 mimic group. The scratch distance of miR-195 simulator group was larger than that of control group. The number of invasive cells in the miR-195 mimic group was significantly lower than that in the control group. The expression of JAK2 protein in miR-195 mimic group was lower than that in miR-NC group. There was a significant negative correlation between the expression level of miR-195 and JAK2 (rhabdomile 0.326 and record 0.00). There are continuous interaction fragments between JAK2 and miR-195. The luciferase activity of miR-195 mimic and wild type JAK2 sequence expression vector was significantly lower than that of wild type JAK2 sequence expression vector.

**Conclusion:**

miR-195 may inhibit the occurrence, metastasis, and invasion of gastric tumor by downregulating the expression of JAK2. miR-195/JAK2 may be a new molecular target for the treatment of gastrointestinal tumors.

## 1. Introduction

Gastric cancer has more than 1 million new cases and about 800000 new deaths every year [1]. The incidence rate of gastric carcinoma is higher in areas with poor living standards, and the incidence in men is about 2 times higher compared to women [2]. Considering that the main pathogenic factor of gastric cancer is Helicobacter pylori infection, promoting living standards and eating habits can slow down [2]. In China, the incidence of gastric carcinoma in rural areas is significantly higher compared to urban residents. This is because China's total population is growing, and the aging rate is increasing [3]. The medical features of gastric carcinoma are anorexia, dyspepsia, weight loss, and abdominal pain, but these symptoms are not obvious in early gastric cancer. Therefore, many cases are not identified with gastric cancer until they are in the late stages. This is also one of the causes of gastric cancerous high-risk to die [4]. Surgical treatment is not only the traditional method for the treatment of gastric cancer but also the only way to cure gastric cancer. With the progress of medical technology, minimally invasive surgery, chemotherapy, targeted therapy, adjuvant, and neoadjuvant therapy have been applied to the treatment of gastric cancer. However, due to the late detection of gastric cancer patients, there is a high metastasis rate, which can easily lead to a poor prognosis; some cases with advanced gastric carcinoma are at poor physical condition and cannot tolerate chemotherapy or surgery; molecular targeted therapy has restrictions on the use of patients who do not express target molecules, or although effective, it is easy to produce drug resistance. Therefore, at present, the overall survival level of patients with gastric cancer is not good. Over the years, many scholars have devoted themselves to the development of new and applicable treatments for gastric cancer.

Many reports have demonstrated the lower miR in a few of tumor tissues [8]. In addition, scholars have suggested that the lower miR-p53 in small cell lung cancer can inhibit cellular metastasis [9]. Moreover, scholars have demonstrated that the expression of miR-195 is also low in gastric cancer [10]. After transfection, the ratio of gastric cancer cells in G 1/G 2 phases increased and that in S phase decreased, suggesting that the overexpression of miR-195 can make gastric cancer cells stay in G1/G2 phase [11]. MicroR transcription NAs is an endogenous noncoding RNA of length 22 nt, which regulates transcription and posttranscriptional gene expression after interacting with target genes. miRNA was first transcribed into an initial transcript of 1000 nt by RNA polymerase II and then cleaved by Drosha enzyme to form a 70 nt miRNA precursor, and finally, a mature miRNA was formed by Dicer enzyme. miR-195 has been shown to suppress replication and speed up cell death in gastric cancer cells by aiming JAK2 [12]. Overexpression of miR-195-5p can inhibit the luciferase activity of JAK2-3′UTR-WT. When the predicted JAK2 binding site is mutated, the inhibitory function of miR-195-5p will disappear, thus confirming that JAK2 is the target of miR-195-5p, and miR-195-5p is also dead in other cancers. Some studies have found that the expression level of miR-195-5p in tumor tissues of patients with esophageal cancer is significantly lower than that in normal tissues. Compared with normal tissues, the expression of miR-195-5p and CDC42 in tumor tissues of patients with esophageal cancer was significantly decreased. The transfection of miR-195 mimics significantly reduced the expression of JAK2 and further inhibited the development of endometrial carcinoma, indicating that miR-195-5p has an inhibitory effect, which may reduce the malignant biological characteristics of endometrial cancer cells by targeting JAK2. The introduction of miR-195-5p mimic into esophageal cancer EC109 and EC9706 cells could significantly upregulate miR-195-5p, downregulate its target gene HMGA2, and inhibit the proliferation of esophageal cancer EC109 and EC9706 cells. The transfection of miR-195 mimics significantly decreased the proliferation activity of Eca109 and TE13 cells and inhibited their clone formation and invasion ability. Studies have shown that miR-195-5p targeting Sox4 can inhibit epithelial-mesenchymal transformation (EMT) of esophageal cancer cells and further inhibit their metastasis and invasion. JAK/STAT pathway is widely involved in cell reproduction, differentiation, transformation, and immune regulation and other biological metabolic processes. In addition, JAK/STAT pathway is also involved in a variety of cellular biological functions in the process of tumorigenesis, such as apoptosis, metastasis, and invasion. JAK inhibitors can selectively inhibit JAK kinase and JAK/STAT pathway as tumor suppressants. The miRNA was low in lung carcinoma, which was related to clinicopathological parameters [13]. JAK kinase (JAKs) is an ancient intracellular protein tyrosine kinase (PTKs) that exists in many organisms. Up to now, four kinds of JAKs, JAK1, JAK2, JAK3, and tyrosine kinase 2 (Tyrosinekinase2, Tyk2), have been identified in mammals. However, the relationship between miR-195, JAK2, and gastric cancer is unclear [14]. The aim is to investigate the relationship between miR-195 and JAK2 in gastric cancer.

## 2. Materials and Methods

### 2.1. Main Reagents, Cell Lines, and Instruments

Gastric cancer MGC803 and NCI tumor N87 cell line are from Shanghai Institute of Life Sciences. miR “195 primer sequence, miR 195mimics, and miR NC control plasmid are from Shanghai Institute of Life Sciences; luciferase reporter gene plasmid containing wild type and mutant JAK2 sequence are from Shanghai Shenggong Biology Co., Ltd.; JAK2 first and second antibodies are from Sigma Co., USA; RNA extraction kit and transfection kit are from Wuhan Bausch Biotechnology Co., Ltd.; MTT Kit is from Wuhan Boshi Biotech Co., Ltd.; luciferase detection kit is from BioVision, USA; Transwell chamber and PCR kit are from Sigma, USA; enzyme labeling instrument is from Shanghai instrument Co., Ltd.; ABI7900PCR amplification instrument is from Shanghai instrument Electric Analytical instrument Co., Ltd.; and flow Cytometer CytoFLEXLX is from Shanghai instrument Electric Analysis instrument Co., Ltd.

### 2.2. Cell Transfection and Grouping

The culture medium of RPMI 1640 was subcultured at 37°C and 5% CO_2_, and the liquid was changed regularly. According to the difference of transfection, the cells were assigned into two groups: miR plasmid NC group (empty plasmid) and miR 195 mimics group (mimic sequence). After transfection, cells continued to incubate for 48 hours.

### 2.3. RT⁃PCR Detection

Expression of miR ‘195 mRNA was isolated by miR Neasy Mini kit (Qiagen China), and the RNA concentration was determined. The qualified total RNA was transcribed into cDNA, and then, PCR amplification was carried out. The results of real-time fluorescence quantitative PCR were expressed by 2^-*Δ*Ct^, noticed in Table 1.

### 2.4. MTT Experiment

The cells of each group were incubated in the plate with 96 wells, and the cell concentration was adjusted to 5 × 10^3^/well. After 24 h incubation, a total of 20 *μ*L MTT solution was supplied into the wells after from 1 day to 5 five days, and the OD value was measured by enzyme labeling instrument after 4 hours of culture. Cell growth inhibited rate (IC) = (1 − OD value of the study group/control group) × 100%.

### 2.5. Cell Migration and Invasion

The cells of each group were digested with trypsin, centrifuged, PBS rinsed 3 times, centrifuged, PBS resuspended, cultured at room temperature for 1 hour, fixed with 75% ethanol for 20 minutes, rinsed 3 times, and incubated at 4°C for 1 h with 10 *μ* LPI under the condition of avoiding light. The fluorescence intensity at Ex = 488 nm was measured by flow cytometry. After centrifugation, Bindingbuffer buffer containing Annexin V-FITC and PI staining solution was added to suspension cells, and 10 min was incubated without light. The apoptosis rate of cells in each group was calculated. Apoptosis rate = number of apoptotic cells/(number of apoptotic cells + number of normal cells) × 100%. Cell migration rate = (0 h scratch area − 24 h scratch area)/0 h scratch area × 100%. The more phase cells of G1/S, the less apoptosis; the more phase cells of G2/S, the more apoptosis.

### 2.6. Transwell Chamber Experiment

The Matrigel matrix glue was diluted with precooled serum-free medium, laid on a 24-well plate, and sterilized by ultraviolet rays. Before use, a small amount of serum-free culture medium was added to incubate for 2 hours of hydration. The specimens were incubated into the plate with 24 wells at a density of 6 × 10^4^ cells/well. RPMI 1640 was added into the lower chamber and incubated for 12 h to wash the dead suspension cells. 4% paraformaldehyde is fixed for 10 min, 0.5% crystal violet staining 10 min. A total of 95% ethanol was rinsed at 4°C for 6 hours. The invasion of 5 visual field cells was evaluated under light microscope, and the average value was taken.

### 2.7. Cell Scratch Test

The cells were inoculated with two straight lines with marker strokes on the back of the orifice plate, the sterile pipette is marked “-” along the cell area, and the scratch area was analyzed under microscope.

### 2.8. Western Blot Detection

JAK2 protein expression removal medium, PBS washing cells, lytic solution to lytic cells, ice bath 30 min 1500 r/min centrifugation 5 min at 40°C, absorption of the upper liquid, ultrasonic nuclear breaking, centrifugation again, and the upper liquid 10 *μ*L were taken out to be tested. Glue, sample, electrophoresis, membrane transfer, membrane cutting, blocking solution for 1 hour, mouse antihuman JAK2 polyclonal antibody, and rabbit antimouse secondary antibodies were marked by horseradish peroxidase. The Bio Rad imager was exposed, and the optical density was measured by ImageLabSoftware.

### 2.9. Experimental Verification of Luciferase

The aiming correlation between miR-195 and JAK2 the wild-type or mutant luciferase reporter gene plasmid vector of JAK2 was transferred into the cells separately according to the steps of the kit, and the culture medium was removed after 48 hours of culture. PBS was rinsed for 3 times, and cell lysate was added. The supernatant was centrifuged for 3 min at 10 min, 40°C and 1000 r/min at 4°C, and the supernatant was taken for luminescence determination.

### 2.10. Statistical Analysis

The experimental results were calculated by SPSS21.0, and measured information (*x* ± *s*) was presented by *t*-test, count data by%, and *χ*2 test between groups. The relation of miR-195 and JAK2 expression was evaluated by Pearson correlation analysis. The difference exhibited is considered to be statistically significant (*P* < 0.05).

## 3. Results

### 3.1. Analysis of the Expression of miRmur195 in Each Group

The level of mi Rmur195 in miR-195-mimics group was higher compared to miR-NC (*P* < 0.05, Figure 1).

### 3.2. Effect of Overexpression of miR-195 on Cell Proliferation and Apoptosis

The cell viability of miR-195 mimics was less compared to miR-NC group (*P* < 0.05, Figure 2). The number of G1 cells in miR-195 mimics was higher than miR-NC, while the cells in G2 phase and S phase were lower compared to miR-NC group. All the data are indicated in Figure 2 and Table 2.

### 3.3. Effects of Overexpression of miR-195 on Cell Migration and Invasion

The scratch distance in miR-195 mimics group was larger compared to miR-NC (*P* < 0.05, Figure 3(a)). The number of cell invasion in miR-195 mimics was less compared to miR-NC, see Figure 3(b).

### 3.4. Effect of Overexpression of miR-195 on JAK2 Protein

The level of JAK2 in miR-195 mimics was weaker than miR-NC (*P* < 0.05), as indicated in Figure 4(b). Pearson correlation analysis indicated that the level of miR-195 m RNA had negative correlation of the level of JAK2 before and after miR-195 mimics transfection, see Figure 4(a).

### 3.5. Prediction and Identification of Downstream Genes of miR-195

Biological information analysis demonstrated there were continuous interplay fragments between miR-195 and JAK2, as indicated in Figure 5(b). The results of luciferase experiment indicated that the luciferase activity of transfected miR-195mimic and wild type JAK2 sequence plasmids was significantly lower compared to wild type JAK2 sequence plasmids alone (*P* < 0.01), see Figure 5(a). The above results indicate that miR-195 directly targets JAK2.

## 4. Discussion

Gastric cancer is a serious neoplasm that develops from the epithelial layer of the stomach. The occurrence of gastric cancer varies significantly by area [15]. The factors of rejuvenation of gastric cancer are dietary changes, work overload pressure, and Helicobacter pylori infection. Gastric cancer can involve any part of the stomach, mostly in the gastric antrum [16]. The large bulk of gastric cancers is adenocarcinomas, which have no classic onset or nonspecific symptomatology like right upper quadrant unpleasantness and belching, most of which are confused with severe gastric diseases are easy to overlook. In China, the percentage of timely identification of gastric cancer is still limited. The pathophysiological phase, position, tissue type, biomedical behavior, and therapeutic interventions of gastric cancer all influence the prognostic value [17]. In China, the infection rate of Hp in adults in areas with great prevalence rate of gastric carcinoma is more than 60% [18]. Helicobacter pylori can increase cancer risk by promoting the conversion of nitrite and nitrosamine; inflammatory process of the gastric epithelium induced by Hp infectious disease and environmental infective factors speeds up the extreme growth of mucosal epithelial cells, giving rise in disordered tumorigenesis; Helicobacter pylori toxic products CagA and VacA may have a carcinogenic effect, and the detection accuracy of anti-CagA [19]. Gastric cancer is a kind of tumor with the participation of multiple genes, which is easy to metastasize in the early stage and has a high degree of malignancy. Therefore, exploring the invasion and expansion is crucial for the management and therapy of tumors.

A variety of miRNA is strongly involved in the carcinogenesis of gastric cancer [14]. MicroRNA (miRNA), a large family of highly conserved RNAs, mainly regulates the level of posttranscriptional gene expression [15]. For example, miR-15a and miR-16-1 are downregulated in most chronic lymphoblastic leukemia and colon carcinoma [16]. miR-155 is strongly upregulated in some cases of Burkitt's lymphoma and several other types of lymphoma. The expression of miR-21 as an inhibitor of apoptosis is increased in glioblastoma cells and tissues. The strong expression of miR-1-03amp107 is correlated to worse outcomes in esophageal squamous cell carcinoma [17]. Therefore, miRNA can provide us with predictive biomarkers for timely identification and prognostic assessment, which can increase our understanding of its role in the occurrence of gastric cancer.

miR-195 is a member of miR-15/107 family and shares common CGACGA-5′ sequence [18]. The hairpin structure of miR-195 leads to its two forms. The coding genes of miR-195-3p and miR-195-5pehsa-miR-195 are located on the chromosome 17p13.1 and induce activation in tumors, cardiac hypertrophy, and schizophrenia. The abnormal regulation of miR-195 is related to many diseases [19]. miR-195 has been demonstrated to be associated with Alzheimer's disease and participates in the pathogenesis of schizophrenia by regulating important brain growth factors. In addition, studies have demonstrated miR-195 shows a significant upregulation in hypertrophic myocardium, and overexpression of miR-195 transgenic mice will eventually lead to heart failure. It is worth mentioning that in many tumors, miR-195 plays a role by targeting oncogenes or tumor suppressor genes and affecting their protein expression, for example, breast, lung, prostate, stomach, bowel, liver, and bladder cancer. miR-195 is located on human chromosome 17. By regulating its target gene, it affects the signal transduction pathway and affects the carcinogenicity of various tumors. For example, miR-195 blocks lung cancer cells in G1 phase by targeting cyclin D3 and promotes lung cancer cell apoptosis by regulating surviving [20]. Studies have demonstrated that the level of miR-195 in serum liver cancer is remarkably lower than the control group, and level of miR-195 in liver cancerous cell line is also lower compared to control THLE-3 cells. Abnormal expression of miR-195 can inhibit the growth, while suppression of miR-195 can increase cancerous growth, suggesting that miR-195 plays the role of suppressor in hepatoma progression. The expression of miR-195 in colorectal cancer is lower compared to normal control group. It represses the growth of colorectal cancerous cells by aiming FGF2 and inhibits proliferation and metastasis of colorectal cancer by targeting WNT3A [21]. The miR-195 was low in AML, and the expression of PTEN and miR-195 were negatively correlated with AML. Other studies have demonstrated that low expression of miR-195 can enhance the invasiveness of breast cancer [22]. Some studies have pointed out that miR-195 levels in gastric cancer patients with lympho-vascular invasion are considerably lower than in patients without distant metastasis. [23]. Therefore, to explore miR-195 in gastric carcinoma and the internal mechanism of regulating cell biological behavior has very important clinical significance to understand tumorigenesis and find specific intervention targets.

JAKs is an ancient intracellular PTKs that exist in many organisms. Up to now, four JAKs, JAK1, JAK2, JAK3, and Tyrosine kinase 2 tyrosine kinases, have been identified in mammals [24]. The primary structure of JAKs consists of FERM domain, SH2 domain, pseudokinase domain, and PTK domain with catalytic activity. JAK/STAT signal pathway is the most widely studied JAKs-mediated signal pathway. STAT is a transcription factor located in the cytoplasm and translocated to the nucleus soon after activation to activate the transcription of the target gene. These STATs, like other transcription factors, have a similar DNA binding domain. In response to the stimulation of up to 50 kinds of cytokines, growth factors, and hormones, JAK/STAT pathway can specifically mediate the expression of different target genes and participate in the regulation of many kinds of life activities in cells. The regulation process is basically the same, to put it simply, JAK catalyzes the phosphorylation of specific tyrosine residues on itself and its receptors by binding to cytokine receptors, thus forming STAT docking sites. STAT is then recruited to bind to and phosphorylate the specific tyrosine residues of STAT. This phosphorylation event leads to the dimerization of STAT, which is rapidly transferred to the nucleus, recognizing the promoter of the target gene and initiating its transcription [24]. JAKs participates in many signal transduction cascades in cells by responding to a variety of growth factors and cytokines and plays an indispensable role in it, so it is particularly important for the negative regulation of JAKs [25]. Current studies have demonstrated that the negative regulation mechanisms of JAK2 kinase are mainly as follows: proteasome-mediated degradation to prevent the continuous activation of JAKs. The activity of JAKs is regulated by protein tyrosine phosphatase (PTPs) dephosphorylation of tyrosine residues involved in the catalytic function of JAKs, and the activity of JAK signal pathway is regulated by cytokine signal inhibitor (SOCS) protein family. Among them, a number of studies have demonstrated that PTPs has made an outstanding contribution to the negative regulation of JAKs. The activation of JAKs family is positively correlated with the phosphorylation of its key tyrosine residues. For example, for JAK2 kinase, the phosphorylation of its Tyr1007 site is necessary to exert its kinase activity, and the mutation at this site will lead to inhibition of JAK2 kinase activity. PTPs can mediate the dephosphorylation of its key sites by binding to JAKs. For example, PTPs SHP-1 containing SH2 domain can mediate its dephosphorylation and inhibit its activity by binding to JAK2 [26].

Since the 20th century, with the deeper of people's understanding of PTKs, it has been gradually found that abnormal activation of PTKs has been detected in proliferative-related diseases such as cancer and leukemia, so tyrosine phosphorylation inhibitors have been developed as potential drugs for treatment [27]. As an important downstream signal pathway in PTKs cells, JAK/STAT signaling pathway takes a key participate in tumor cells and tumor microenvironment. JAK and STAT3 are generally believed to be important targets for cancer therapy [28]. Persistent activation of JAK/STAT pathway can be detected in bone marrow proliferative tumors, glioblastoma, thyroid cancer, and other cancers. Among them, the most widely studied is the relationship between JAK/STAT signaling pathway and myeloproliferative tumors and the development of this pathway inhibitor to effectively treat the disease [29]. As early as 2005, some scholars found that there was a JAK2V617F mutation or exon 12 mutation in myeloproliferative tumors, which provided a genetic basis for the continuous activation of JAK/STAT signal in patients with MPN. In view of this, a variety of JAK inhibitors have been developed, and two compounds ruxolitinib and fedratinib have entered the clinical stage. However, the currently developed inhibitors have no choice for mutants of JAKs, so they not only interfere with JAK mutants but also disturb the normal JAK/STAT signal pathway. Growth hormone (GH) and prolactin are involved in the proliferation, differentiation, and survival of mammary epithelial cells by activating JAK2 kinase and regulating its downstream transcription factor STAT5. The imbalance of JAK2-STAT5 activity can lead to breast developmental diseases, including breast cancer. In this process, the normal operation of JAK2-STAT5 signal transduction pathway depends on crosstalk with other signal transduction pathways. For example, Akt1 increases the expression of Akt1 and phosphatidylinositol-3-phosphate (PI3K) subunits by activating STAT5 phosphorylation and further regulates the activity of PI3K by combining with it, which means that there is a strong tandem between PI3K-Akt and JAK2/STAT5 signal pathways. Related studies also found that ERK1/2 was also significantly activated in overexpressed constituent activated STAT5 cells, which means that there may be a close relationship between MAPK/ERK signaling pathway and JAK/STAT pathway (Nyga et al. 2005). More studies have demonstrated that JAK2 kinase can participate in the regulation of cell survival and apoptosis by mediating the expression of antiapoptotic cell death factor Bcl-XL. In some hematological malignancies, JAKs is often abnormally activated. Transforming growth factor-*β* 1 (TGF-*β* 1) can upregulate STAT3 phosphorylation by activating JAK/STAT3 signal pathway, induce mesenchymal stem cells (MSCs) to differentiate into cancer-related fibroblasts (CAFs), and enhance the migration and invasion ability of rectal cancerous cells. In addition, there is ample evidence that JAK/STAT signal imbalance is an important driver of drug resistance in glioblastoma (GBM) [32]. The continuous activation of STAT3 caused by JAK/STAT signal imbalance substantially enhances a variety of tumorigenic functions of GBM, including cell proliferation, antiapoptosis, angiogenesis, stem cell maintenance, and immunosuppression. In summary, the development of a wide range of JAK/STAT signal pathway inhibitors is far from enough, for different diseases, due to different pathogenesis or different STATs activated downstream of JAKs, it is necessary to develop targeted inhibitors, which requires further exploration and clinical data and has a broad research prospect.

In this study, we constructed a stable overexpression miR-195 vector in vitro and confirmed that the transfection efficiency was satisfactory after transfection of gastric cancer cells. The level of miR-195 in miR-195-MIMICS group was significantly higher than that in miR-NC group. The cell survival rate of miR-195 mimic group was lower than that of miR-NC group (*P* < 0.05). Compared with miR-NC group, the number of cells in G1 phase increased, the cells in G2 phase and S phase decreased, and the proportion of cells in G2 and S phase decreased in miR-195 mimic group. The scratch distance of miR-195 simulator group was larger than that of control group. The number of invasive cells in the miR-195 mimic group was significantly lower than that in the control group. The expression of JAK2 protein in miR-195 mimic group was lower than that in miR-NC group. There was a significant negative correlation between the expression level of miR-195 and JAK2 (rhabdomile 0.326 and record 0.00). There are continuous interaction fragments between JAK2 and miR-195. The luciferase activity of miR-195 mimic and wild type JAK2 sequence expression vector was significantly lower than that of wild type JAK2 sequence expression vector. Further studies indicated that the proliferation, invasion, and migration ability of tumor cells transfected with miR-195 decreased, suggesting that there is a certain relationship between miR-195 and gastric cancer, which is basically consistent with other research results [16]. miR-195 follows the characteristics of miRNAs in eukaryotic cells, that is, it binds to the specific sites of transcriptional genes and silences transcriptional gene translators, resulting in different biological effects, that is, inhibiting the proliferation of gastric cancer cells, promoting apoptosis, and realizing the self-metabolism of tumor cells [17]. The chemokine family members closely related to gastric cancer are CXC, CC, and CX3C subtypes and their corresponding receptors, which promote the proliferation, invasion, and metastasis of gastric cancer cells [18]. Some chemokines can also induce drug resistance or drug resistance mutations in tumor cells, affect the effect of tumor chemotherapy, and mediate the activation of multiple signal pathways such as rapamycin target protein (mTOR) and JAK/STAT [19, 20]. Chemokine 5 belongs to the small molecular cytokine protein family, which can recruit a large number of immune cells, such as T lymphocytes, antigen presenting cells, and inflammatory cells, such as neutrophils, macrophages, and fibroblasts [21]. And then release a large number of inflammatory factors to produce a microenvironment conducive to tumor cell proliferation and invasion and inhibit apoptosis. Inducing neovascularization to provide nutrition for malignant proliferation of tumor cells; meanwhile, it can mediate immune escape to reduce the monitoring of the immune system or increase the molecular variation on the cancer cellular surface to avoid recognition by antigen presenting cells [22–25]. One study reported the both of CCL5 and CCR5 can increase the invasive ability of salivary adenoid cystic carcinoma (SACC) cells. Liang et al.'s study indicated that serum CCL5 level in patients with clear cell carcinoma was greater compared to normal people and was closely related to the clinicopathological features and prognosis of patients [26]. In addition, scholars have found that CCL5 can downregulate miR-200b to promote EGFR-dependent angiogenesis and VEGF synthesis in human chondrosarcoma [27]. miR-195 follows the characteristics of miRNAs in eukaryotic cells, that is, it binds to the specific sites of transcriptional genes and plays the role of silencing transcriptional gene translation proteins, resulting in different biological effects [28]. Online biological information analysis indicated that JAK2 was the downstream targeting gene of miR-195. Correlated assessment indicated a negative correlation existed between miR-195 overexpression group and control group. Luciferase assay further confirmed that miR-195 straightly aimed JAK2. The reason may be that miR-195 decreased JAK2 and then regulates the biological events of gastric cancer.

In summary, this study suggests that miR-195 may inhibit the progression of gastric cancer by reducing JAK2, and miR-195/JAK2 may be the biochemical target of anticancer drugs for gastric cancer. There are also some shortcomings in this study. We have not studied other target genes and related pathways. In the future research, we will increase the study of other target genes and related pathways to further explore the biochemical targets of gene therapy for gastric cancer.

## Figures and Tables

**Figure 1:** Note: the relative level of miR-195 mRNA in mi R-NC group was compared with that in miR-195 mimics group (*P* < 0.05). ∗ indicates that the difference is statistically significant (*P* < 0.05).

**Figure 2:** Note: (a) MTT test detected the capability of cell proliferation after miR-195 mimics transfection. (b, c) The apoptosis after miR-195 mimics transfection by flow cytometry, the ratio of G1/S and G2/S phase cells. The apoptosis rate of mi R-NC group was remarkably greater than miR-195mimics group. ∗Compared with miR-195 mimics group, *P* < 0.05.

**Figure 3:** Note: (a) scratch distance of each group (100×). (b) The number of cells attached to the bottom of the membrane in each group (100×). ∗Compared with miR-NC group, *P* < 0.05.

**Figure 4:** Note: (a) miR-195 has negative correlation with JAK2. (b) The content of JAK2 protein in cells of each group. ∗Compared with miR-NC group, *P* < 0.05.

**Figure 5:** Note: (a) double luciferase report results; prediction map of targeted binding sites of (b) miR-195 and JAK2. ∗∗Compared with JAK2 5WT group, *P* < 0.01.

**Table 1:** Primer sequence.

Genes	Upstream primer	Downstream primer
miR-195	5′⁃ATAACCTACCAGCGCCGAATTCGGGACCA⁃3′	5′⁃ACCACCGACTTGTGACA⁃3′
U6	5′⁃TATTGACATTAGTTAAT⁃3′	5′⁃TTTAGAAGACTCCCTAGAGTA⁃3′

**Table 2:** The number of cells in G1, G2, and S phases in each group by flow cytometry (%).

Group	miR-NC	miR-195 mimics
G1	69.43 ± 11.55	84.68 ± 12.66
G2	4.46 ± 0.42	0.01 ± 0.07
S	25.91 ± 2.31	12.95 ± 3.53

## Data Availability

No data were used to support this study.

## References

[1] Liang M., Huang G., Liu Z. (2019). Elevated levels of hsa circ 006100 in gastric cancer promote cell growth and metastasis via miR-195/GPRC5A signalling. *Cell Proliferation*.

[2] Lin X., Wang S., Sun M. (2019). miR-195-5p/NOTCH2-mediated EMT modulates IL-4 secretion in colorectal cancer to affect M2-like TAM polarization. *Journal of Hematology & Oncology*.

[3] Gao K., Wu J. (2019). National trend of gastric cancer mortality in China (2003–2015): a population-based study. *Cancer Communications*.

[4] Wei L., Han C., Wang D. (2021). Protective role of astragaloside IV in gastric cancer through regulation of miRNA-195-5p-mediated PD-L1. *Immunopharmacology and Immunotoxicology*.

[5] Panpan Z., Xiong S., Meng C. (2021). Micro-RNA-195 inhibits the dry characteristics and invasive ability of CD44~+ gastric cancer stem cells. *Jiangsu medicine*.

[6] Sui H., Zhu C., Li Z., Yang J. (2020). Propofol suppresses gastric cancer tumorigenesis by modulating the circular RNAPVT1/miR1955p/E26 oncogene homolog 1 axis. *Oncology Reports*.

[7] Chen C., Xiaotong Z., Xu Y. (2021). Propofol prevents the aggressive progression of oral squamous cell carcinoma via regulating circ_0005623/miR-195-5p/HOXB7 axis. *Biotechnology and Applied Biochemistry*.

[8] Song W., Cui Z., Liu H., Xue L., Ju H. (2020). The expression and prognostic value of miR-195-5p in patients with advanced gastric cancer after chemotherapy. *Journal of BU ON.: Official Journal of the Balkan Union of Oncology*.

[9] Yan Y., Zheng L., Du Q. (2021). Interferon regulatory factor 1 (IRF-1) downregulates checkpoint kinase 1 (CHK1) through miR-195 to upregulate apoptosis and PD-L1 expression in hepatocellular carcinoma (HCC) cells. *British Journal of Cancer*.

[10] Youjing T., Hao Z., Xingchao C., Jun L., He L. (2020). Mechanism of mir-195-5p targeting hmbox1 regulating proliferation, migration, invasion and apoptosis of gastric cancer cells. *Chinese Journal of Gerontology*.

[11] Nie H., Mu J., Wang J., Li Y. (2018). miR1955p regulates multidrug resistance of gastric cancer cells via targeting ZNF139. *Oncology Reports*.

[12] Wu Z. (2021). miR-195 connects lncRNA RUNX1-IT1 and cyclin D1 to regulate the proliferation of glioblastoma cells. *The International Journal of Neuroscience*.

[13] Wang G., Wang H., Zhang L., Guo F., Wu X., Liu Y. (2021). miR-195-5p inhibits proliferation and invasion of nerve cells in Hirschsprung disease by targeting GFRA4. *Molecular and Cellular Biochemistry*.

[14] Xiaoting Z. (2020). Expression of serum miR-200c-3p and miR-195-5p in ovarian cancer and its prognostic value. *Laboratory medicine and clinic*.

[15] Yan B., Ren Z., Sun J., Ding C., Yang D. (2020). IGF2-AS knockdown inhibits glycolysis and accelerates apoptosis of gastric cancer cells through targeting miR-195/CREB1 axis. *Biomedicine & Pharmacotherapy*.

[16] Mu L., Yang F., Guo D., Li P., Zhang M. (2020). Overexpression of secretory clusterin (sCLU) induces chemotherapy resistance in human gastric cancer cells by targeting miR-195-5p. *Bioengineered*.

[17] Zou J., Liao X., Zhang J., Wang L. (2019). Dysregulation of miR-195-5p/-218-5p/BIRC5 axis predicts a poor prognosis in patients with gastric cancer. *Journal of Biological Regulators and Homeostatic Agents*.

[18] Liu W., Chen H., Wang D. (2021). Protective role of astragaloside IV in gastric cancer through regulation of microRNA-195-5p-mediated PD-L1. *Immunopharmacology and Immunotoxicology*.

[19] Qian Y., Lizhen C., Li Y., Liqi L., Yuanshuai H. (2020). Study on the expression and clinical significance of miR-195 in gastric cancer based on bioinformatics. *Labeled Immunoassay and Clinical*.

[20] Tong K. H., Qian J. (2021). Long non-coding RNA FGD5-AS1 is an inducer of cisplatin chemoresistance in gastric cancer cells by sponging miR-195. *Journal of Biological Regulators and Homeostatic Agents*.

[21] Jing H. (2020). *miR-195 Inhibits the Proliferation of Esophageal Cancer Cells through Targeted Regulation of Cyc Hin D 1 and Cdc42*.

[22] Chen Z., Licui Z., Zhu M. (2020). MiR-195-5p targeted regulation of ELMO2 to inhibit IL-17-induced invasion and migration of gastric cancer cell line AGS. *Chinese Journal of Immunology*.

[23] Yang Y., Wu F., Zhang J. (2019). EGR1 interacts with DNMT3L to inhibit the transcription of miR-195 and plays an anti-apoptotic role in the development of gastric cancer. *Journal of Cellular and Molecular Medicine*.

[24] Ye R., Wei B., Li S. (2017). Expression of miR-195 is associated with chemotherapy sensitivity of cisplatin and clinical prognosis in gastric cancer. *Oncotarget*.

[25] Huang B., Chang C., Wang B. L., Li H. (2019). ELK1-induced upregulation of lncRNA TRPM2-AS promotes tumor progression in gastric cancer by regulating miR-195/ HMGA1 axis. *Journal of Cellular Biochemistry*.

[26] Liu X., Pu K., Wang Y., Chen Y., Zhou Y. (2021). Gastric cancer-associated microRNA expression signatures: integrated bioinformatics analysis, validation, and clinical significance. *Annals of Translational Medicine*.

[27] Zhao D.-L., Wu Q.-L. (2019). Effect of inhibition to yes-related proteins-mediated Wnt/*β*-catenin signaling pathway through miR-195-5p on apoptosis of gastric cancer cells. *European Review for Medical and Pharmacological Sciences*.

[28] Wang C.-Q. (2019). miR-195 reverses 5-FU resistance through targeting HMGA1 in gastric cancer cells. *European Review for Medical and Pharmacological Sciences*.

[29] Wang J., Li L., Jiang M., Li Y. (2017). MicroRNA-195 inhibits human gastric cancer by directly targeting basic fibroblast growth factor. *Clinical and Translational Oncology*.

[30] Shen Y. H., Xie Z. B., Yue A. M. (2016). Expression level of microRNA-195 in the serum of patients with gastric cancer and its relationship with the clinicopathological staging of the cancer. *European Review for Medical and Pharmacological Sciences*.

[31] Zhang W., Wang Y., Zhu Z., Zheng Y., Song B. (2018). Propofol inhibits proliferation, migration and invasion of gastric cancer cells by up-regulating microRNA-195. *International Journal of Biological Macromolecules*.

[32] Wang F., Ruan L., Yang J., Zhao Q., Wei W. (2018). TRIM14 promotes the migration and invasion of gastric cancer by regulating epithelialtomesenchymal transition via activation of AKT signaling regulated by miR1955p. *Oncology Reports*.

